The article "Application of Absorbable Suture in Strabismus Correction and Nursing Management Advantage of Watson Care Theory in Perioperative Period" was retracted in 2023. Reasons: unreliable results or conclusions; concerns about the data; concerns about the peer review; concerns about the citations.

# Application of Absorbable Suture in Strabismus Correction and Nursing Management Advantage of Watson Care Theory in Perioperative Period

**DOI:** 10.1155/2022/8739551

**Published:** 2022-03-04

**Authors:** Weina Guo, Suling Yang, Yuexing Gong, Lizhi Zhang, Tao Jin, Jiancang Wang, Xiting Guo, Huihui Sun, Yanxia Song, Haixia Tian

**Affiliations:** ^1^Department of Ophthalmology, Bethune International Peace Hospital, Shijiazhuang, 050082 Hebei, China; ^2^Department of Ophthalmology, Children's Hospital of Hebei Province, Shijiazhuang, 050000 Hebei, China; ^3^Department of Nursing, Shijiazhuang Medical College, Shijiazhuang, 050000 Hebei Province, China

## Abstract

**Objectives:**

The article is aimed at investigating the suture effect of absorbable suture in strabismus correction and the advantage of Watson care theory.

**Methods:**

148 children with strabismus were enrolled in this study and divided into two groups. The control group received routine nursing, and on this basis, the observation group was given Watson care theory nursing and eye muscle suture with absorbable sutures. The degree of cooperation (induction compliance checklist (ICC) score), negative emotion (modified Yale preoperative anxiety scale (m-YAPS) score), pain (face pain scale (FPS) score), quality of nursing management, parents' satisfaction, clinical efficacy, and adverse reactions were compared.

**Results:**

After nursing and surgical treatment, all children's strabismus symptoms were improved, and the improvement of strabismus and visual function in the observation group was more obvious. Watson care nursing can effectively improve the nursing management quality, parents' satisfaction, children's negative emotions, and treatment compliance.

**Conclusions:**

As a result, Watson care theory nursing is of great significance for improving the relationship between nurses and patients and building a harmonious hospital.

## 1. Introduction

Strabismus, with a high incidence rate of about 1.2%-3.15%, is accepted as a common disease among children in China [1]. The main performance of strabismus is eye movement disorder, which will further affect visual function; if not corrected in time, it will lead to amblyopia and fusion dysfunction and cause its appearance defects [2], which will cause adverse effects on the quality of life and psychology of children. Preschool is the stage of children's mental maturity, and their ability to bear pressure is weak; if their personal emotions are affected by strabismus, or they are rejected and alienated by other playmates in life, it will further affect the healthy development of their personal mind [3]. Therefore, early surgical correction of strabismus in children, for its subsequent recovery, as well as the healthy development of the mind, has important significance. Children are generally afraid of hospitalized surgical correction, and because of their weak ability of psychological adjustment and tolerance [4], it is easy to affect the compliance of hospitalized treatment and then influence the effect of surgical treatment. However, due to the lack of equal treatment and spiritual communication in children's nursing process, it is easy to cause children's panic and aggravate the contradiction between nurses and their patients. Therefore, we explore a new nursing model in the perioperative nursing of strabismus children, so as to improve the cooperation of surgical treatment and rehabilitation exercise and the surgical effect.

Nursing is developing constantly, and the nursing technology and the types of nursing materials are constantly updated and improved, and so is the concept of nursing. The concept of patient-oriented nursing is continuously implemented in the daily service, aiming at providing better quality service for patients [5]. Caring is the core of nursing care in the theory of Watson care; in the daily nursing process, the nurses should take “respect” as the connotation and “concern” as the driving force, which will help to build a harmonious medical environment [6] and improve patient's treatment experience and recovery. Especially for children with strabismus, because their mental development is not mature enough and they live in a strange medical environment, they are prone to panic and anxiety [7]. Therefore, it is of great significance for clinical treatment and postoperative rehabilitation to uphold Watson's “human text” nursing concept and carry out individualized nursing for each child.

In this study, the suture used in strabismus surgery also has a great impact on the postoperative rehabilitation. Human eyes are extremely sensitive; as a kind of foreign body, suture can easily lead to immune rejection. In addition to causing foreign body sensation, it can also lead to the accumulation of related inflammatory factors, infection, and even scar formation. Therefore, the texture of suture is of great significance for the surgical efficacy and postoperative rehabilitation of children [8]. In this study, 6-0 absorbable suture produced by the Johnson Company of USA was selected as suture, with the characteristics of low friction coefficient and self-absorption [9, 10], which can reduce the pain or secondary trauma caused by suture removal. However, it also has corresponding disadvantages, such as the local mechanical reaction is slightly larger, and the firmness of suture knot is also reduced to a certain extent [11, 12]. Therefore, the clinical effect of absorbable suture in the strabismus correction, and the advantages of Watson care theory in perioperative nursing care of children with strabismus are studied.

## 2. Materials and Methods

### 2.1. Materials

#### 2.1.1. The Choice of Research Object

148 children with strabismus treated in the Bethune International Peace Hospital from January 2018 to January 2020 were chosen as the subjects investigated. All children and their guardians who participated in the study gave informed consent to the study and voluntarily signed informed consent. This study was approved by the Ethics Committee of Bethune International Peace Hospital. Inclusion criteria: (1) strabismus was diagnosed according to the criteria in *Esotropia and Exotropia Preferred Practice Pattern* [13]; (2) age range: three to seven years old; (3) received strabismus surgery; (4) clinical cooperation can be combined with various clinical examinations. Exclusion criteria: (1) combined with amblyopia; (2) combined with eye infection, such as keratitis and conjunctivitis; (3) previous eye surgery; (4) combined with high refractive error, anisometropia was more than 2.5D; (5) combined with myasthenia gravis.

#### 2.1.2. Absorbable Suture

The absorbable suture was purchased from the Johnson Company of USA; the specification was 6-0 round needle suture (Figure 1). The absorbable suture was made of polyglycolic acid, which could be self-degradable and absorbed in the tissue. It had the characteristics of fast absorption, small stimulation, and light foreign body reaction. It could effectively avoid the secondary injury caused by suture removal. In the observation group, after the corresponding ophthalmic muscles were severed during the operation, the muscles were retreated or shortened according to patient's condition, and then, the absorbable suture was used for anastomosis.

### 2.2. Methods

#### 2.2.1. Group and Treatment Plan Design

148 children with strabismus were divided into control group and observation group, with 74 cases in each group. In the process of strabismus surgery, proline nonabsorbable suture and golden ring absorbable suture were used, respectively. At the same time, routine nursing was conducted in the control group during the perioperative period, and the children in the observation group were given Watson care.

#### 2.2.2. Watson Care Implementation Plan

Watson nursing care group was established, with the director of nursing department and department director as the team leader. The team members included one head nurse, three nurses in charge, and five nurses. The team leader should train the team members, so as to change the nursing concept of nurses. It is necessary to educate people-oriented, think about problems from the perspective of patients, think about patients everywhere, and establish the consciousness of active service for patients. At the same time, clinical practice can help nurses better grasp the connotation of human care and instill trust and hope into patients.

Before the operation, health education was undergone through PPT, short video of medical animation, brochures, and so on, so as to vividly tell the children and their parents about the clinical manifestations and surgical treatment of strabismus. Moreover, it can explain the surgical process to the children step by step in the mode of game breakthrough, so as to increase the understanding of parents and children about the treatment of strabismus; psychological care is an important part of humanistic care; nurses should change their role concept, help children to receive medical treatment, listen to their voices in time, and pay attention to their emotional changes, so as to better understand their mentality and improve children's ability to handle disease objective to improve the acceptance of surgical treatment and enhance their confidence to overcome the disease; in terms of the layout of humanistic care environment, the sunny room is selected as the ward, and the color of the room is set as pink. Warm color can give children more sense of protection. Children's paradise is set up to give children more space to communicate with each other and reduce their fear. At the same time, the hospital bed is equipped with fence to prevent the occurrence of children falling out of bed.

During the operation, contact the operating room nurses, clinical support center, and anesthesiologists to do a good job in the operation table of children and give priority to the younger children to accept the operation, and the children who have been on the same stage for a long time should be supplemented with water and electrolyte through infusion; during the transfer and operation, the limbs of the children should be covered with insulation blanket to keep warm, the temperature of the operating room should be controlled at about 28°C, and all the flushing liquid needed in the operation should be heated to 37°C in the incubator; in terms of anesthesia intervention, nurses had introduced the anesthesia process in the ward through game breakthrough. At the same time, the anesthesiologist could also transfer the attention of the children by playing relaxed music and given them some physical actions such as caressing and holding hands, so as to give them encouragement and comfort.

After the operation, the nurses should do a good job in postoperative flexible nursing, guide the time of eating and drinking water, and introduce the completion of the operation to the parents with the doctor to relieve their tension; in terms of rehabilitation training, the visual perception training method was used to guide children's postoperative rehabilitation exercise, and according to the degree of illness and postoperative examination results of each child, a special exercise program was set for the adjustment, and the exercise video was sent to WeChat group, which was convenient for parents to guide children's rehabilitation exercise; after discharge, follow-up work outside the hospital was done, and the results of rehabilitation training were followed up in time. At the same time, the review results of children would be arranged into electronic documents every week, so as to better guide children to carry out rehabilitation exercise.

#### 2.2.3. Assessment Tools and Assessment Methods

1. Induction compliance checklist (ICC) was used to evaluate the degree of cooperation between the two groups during anesthesia induction [14]. There are 11 items in the scale. The higher the score, the lower the degree of cooperation during anesthesia induction
2. The modified Yale preoperative anxiety scale (m-YPAS) was used to describe the perioperative psychological anxiety of children [15]. In the scale, 22 items were included to evaluate children's anxiety state from the aspects of children's activities, language, emotion, awakening, and dependence on their parents. Most items were scored at level six, and a few items were scored at level four, with a total score of 23-100. The higher the score, the more obvious the anxiety state
3. Face pain scale (FPS) was used to evaluate the postoperative pain of children [16]. The facial expressions of children were compared with six different facial expressions in smiley face scale, so as to score the pain degree of children. The higher the score, the more obvious the pain degree
4. Self-designed satisfaction scale was used to assess the family satisfaction, mainly evaluated in terms of service attitude, surgical quality, psychological intervention, medical environment, and ward management, and each index was scored at level four; the higher the score, the more satisfied the patients were
5. Perioperative management quality was evaluated from the standard rate of admission education, preoperative interview, surgical handover, surgical punctual opening, and rehabilitation guidance
6. Clinical efficacy evaluation: the distance and near strabismus of the children were detected by triple prism combined with occlusion method before operation, and at the first and third month after operation, and the detection results were expressed by prism degree (Δ). The visual function recovery of children was divided into I, II, and III levels, which were simultaneous vision, fusion vision, and stereopsis. All the tests were conducted by two senior ophthalmologists

#### 2.2.4. Statistical Methods

SPSS18.0 statistical software package was used for data analysis, descriptive statistical analysis, and nonparametric test analysis. *P* < 0.05 was considered statistically significant.

## 3. Results and Discussion

### 3.1. Effect Picture of Eye Position before and after Strabismus Correction

The two cases chosen were both exotropia; after surgical correction and postoperative rehabilitation training, their appearance had been significantly improved, the eyes position were both in the positive position, and the clinical effect was obvious (Figure 2).

### 3.2. Management Quality in Perioperative Period

The effect of perioperative management played a significant role in the treatment compliance and mentality of children. This study evaluated the management quality of nursing staff during perioperative period from admission education, preoperative interview, surgical handover, surgical punctual opening, and rehabilitation guidance. After the statistical questionnaire, it was found that the management quality of observation group was higher (*P* < 0.05) (Figure 3).

### 3.3. Cooperation, Anxiety, and Pain of Children in Perioperative Period

Perioperative treatment compliance of children was of great significance to improve the success rate of surgery and treatment effect. By comparing the m-YAPS score of the two groups, the treatment compliance of children in the observation group was better (*P* < 0.05) (Figure 4(a). During the perioperative period, due to the young age and immature mental development of the children, the emotional control was of great significance for the treatment of themselves and other children. According to the research, the ICC score of the control group was higher (*P* < 0.05), which indicated that the emotional fluctuation was more obvious during the perioperative period, and it was easier to produce anxiety and depression (Figure 4(b). Postoperative pain was the key to affect the emotion of children and their parents and also an important aspect of humanistic care. The research found that the FPS scores in the control group were higher (*P* < 0.05), which indicated that the postoperative pain was server (Figure 4(c).

### 3.4. Incidence of Postoperative Adverse Events after Strabismus Surgery

Due to the foreign body reaction of suture and poor wound healing, it was easy to cause postoperative adverse reactions. The study found that the incidence of adverse reactions such as photophobia, tears, scleral scar, conjunctival granuloma, pain, and foreign body sensation in the observation group was significantly lower (*P* < 0.05) (Figure 5), indicating that the postoperative wound suture reaction was relatively light, and the recovery was better.

### 3.5. Changes of Strabismus and Visual Function

In this study, the treatment effect was evaluated mainly by the changes of children's near and far strabismus before and after treatment, as well as the changes of the number of children with grade I, II, and III visual function. At the 3rd and 6th month after operation, the strabismus degree of the two groups decreased significantly, especially in the observation group (Figures 6(a) and 6(b)). In terms of visual function, difference was not found in the proportion of grade 3 visual function between the two groups on the 7th day after treatment (*P* > 0.05). At the 1st and 3rd month after treatment, the visual function of the two groups was significantly improved, and the proportion of grade 3 visual function in the observation group was significantly higher (*P* < 0.05) (Figure 6(c)).

### 3.6. Family Members' Satisfaction with Nursing

Perioperative nursing satisfaction was the most real evaluation of the nursing effect of nurses. This study evaluated the service quality of nursing staff from the aspects of service attitude, surgical quality, psychological intervention, medical environment, and ward management. After the questionnaire survey, we found that the service quality of the observation group was significantly higher (*P* < 0.05) (Figure 7), which indicates that its nursing satisfaction was higher.

## 4. Discussion

In clinical treatment, nursing staff not only need to cooperate with doctors to do a good job in the infusion treatment of patients but also shoulder the daily nursing work of patients, which plays an irreplaceable role in the recovery process of patients' condition. Therefore, improving the quality of clinical nursing plays an important role in improving the prognosis of patients and their medical experience. Besides the technical level, the renewal of nursing concept is also the key point to improve the quality of nursing. In the process of child care, “people-oriented” is the core concept of nursing; more patience and care are needed [17], only by fully understanding the cultural background of children and their parents, respecting the values of children, and meeting the personalized needs of different children can we better build a harmonious nurse patient relationship. Watson theory believes that nursing work is a discipline of nurses' sincerity, care, and love [18]. In the process of service, fully reflecting the humanistic concern is of great significance for nurses to get occupation identity, and it is an indispensable structural factor in high-quality nursing. Therefore, the role of Watson care in improving the quality of care could not be ignored.

In this study, in order to quantitatively evaluate the quality of Watson care during perioperative period, we designed the perioperative management quality score scale, which evaluated the management quality from admission education, preoperative interview, surgical handover, surgical punctual opening, and rehabilitation guidance. After Watson care physiotherapy guidance and training, nurses fully improved the standardization and quality of nursing operation from all aspects during perioperative period, such as adopting diversified modes of admission education, using warm color painting in ward, setting up children's paradise, reasonably arranging operation, and conducting rehabilitation training guidance and follow-up after operation [19]. Through the above measures, the people-oriented concept was implemented in the whole process of treatment and recovery. Therefore, the quality of perioperative management in the observation group was greatly improved.

Children's fear of strange environment and surgery will greatly affect the treatment of strabismus [20]; as a result, reducing their fear and improving the level of cooperation during anesthesia induction are of great significance for the smooth operation and avoiding the occurrence of adverse psychological stress. In Watson care, it is very important to establish a relationship of help and trust with patients and help patients reduce negative emotions [21]. Through professional psychological counseling and attention to the emotional changes of children, problems will be found, and psychological counseling will be conducted in time. At the same time, the establishment of children's playroom can increase the opportunity of communication between children, let children communicate and play freely, and reduce their fear of strange environment. Gürcan and Atay Turan [22] found that Watson theory care nursing could provide humanistic and compassionate care for cancer children and provide a good nursing environment for their rehabilitation, which is consistent with this study. Moreover, in order to avoid the anxiety and fear during anesthesia induction, the nurses led the children to gradually get familiar with the operation process in the mode of breakthrough game before operation and arranged the reception time reasonably [23], so as to avoid hunger and thirst to increase their fear and anxiety. Therefore, the cooperation degree of anesthesia induction and positive emotion in the observation group were effectively improved.

During strabismus surgery, the cutting and pulling of the eye muscle and the stimulation of the suture will cause a series of adverse stimulation reactions to the eyes, while children's tolerance for pain and discomfort is weak, and the discomfort of the eyes will be further magnified after operation [24]. The absorbable suture used in the observation group had low friction coefficient and relatively little irritation to the eye suture [25], which could better reduce the postoperative intraocular foreign body sensation and the occurrence of photophobic tears. At the same time, its absorbability could avoid the secondary injury brought by suture removal and reduce the pain of children. Therefore, the pain events in the observation group decreased significantly. However, absorbable suture is easy to cause the accumulation of inflammatory cells, and its slow absorption process will lead to a relatively long duration of chronic inflammation, which will increase the incidence of conjunctival granuloma and scleral scar [26]. In summary, absorbable suture could effectively reduce the occurrence of adverse eye irritation in children, so as to significantly improve the surgical efficacy. At the same time, benefit from better follow-up after strabismus surgery, as well as detailed rehabilitation training guidance during the follow-up period, could promote the recovery of children's visual function [27]. Therefore, strabismus degree and visual function in the observation group was greatly improved, which significantly improved satisfaction of children's parents, better improve the medical relationship, and build a harmonious hospital.

## 5. Conclusion

In this study, through Watson care course training for nursing staff, the “people-oriented” nursing concept of nursing staff was effectively improved. In the process of nursing, nurses take care as the core and start from the perspective of children, which effectively reduce the negative emotions of children and improve their treatment compliance and nursing management quality as a whole. At the same time, the use of absorbable suture can reduce the occurrence of eye adverse events and improve the clinical efficacy. Therefore, Watson care theory plays a great role in improving patients' satisfaction and relationship between nurses and patients and building a harmonious hospital. However, in this study, we did not set up a blank control group using absorbable suture alone, and the study sample size was small, which may offset the results. The above aspects should be improved in the follow-up study.

## Figures and Tables

**Figure 1:** Appearance design of absorbable suture.

**Figure 2:** Eye position change map before and after treatment in children with strabismus (a, b).

**Figure 3:** The comparison of perioperative management quality in terms of preoperative interview, surgical handover, surgical punctual opening, and rehabilitation guidance.

**Figure 4:** The comparison of treatment compliance (m-YPAS score) (a), negative emotion (ICC score) (b), and postoperative wound pain (FPS score) (c).

**Figure 5:** The comparison of postoperative adverse reactions in terms of photophobia, tears, scleral scar, conjunctival granuloma, pain, and foreign body sensation.

**Figure 6:** Comparison of near strabismus (a), far strabismus (b), and visual function (c) between the two groups after operation and rehabilitation training, ^∗^*P* < 0.01.

**Figure 7:** The comparison of satisfaction degree in terms of service attitude, surgical quality, psychological intervention, medical environment, and ward management.

## Data Availability

The labeled dataset used to support the findings of this study are available from the corresponding author upon request.

## References

[1] He H., Fu J., Meng Z., Chen W., Li L., Zhao X. (2020). Prevalence and associated risk factors for childhood strabismus in Lhasa, Tibet, China: a cross-sectional, school-based study. *BMC Ophthalmology*.

[2] Beisse F., Koch M., Uhlmann L., Beisse C. (2020). Consideration of eyeball length and prismatic side-effects of spectacle lenses in strabismus surgery-a randomised, double-blind interventional study. *Graefe's Archive for Clinical and Experimental Ophthalmology*.

[3] Kitasato M., Iwamitsu Y., Iwata Y., Ueta T., Fukaya E., Ishikawa H. (2020). Investigation of stress and distress experienced by guardians of children with strabismus and/or amblyopia. *Journal of Binocular Vision and Ocular Motility*.

[4] Jin Y., Jiang A., Jiang W. (2021). Self-produced audio-visual animation introduction alleviates preoperative anxiety in pediatric strabismus surgery: a randomized controlled study. *BMC Ophthalmology*.

[5] Murali K. P. (2020). End of life decision-making: Watson's theory of human caring. *Nursing Science Quarterly*.

[6] Durgun Ozan Y., Duman M., Çiçek Ö., Baksi A. (2020). The effects of clinical education program based on Watson's theory of human caring on coping and anxiety levels of nursing students: a randomized control trial. *Perspectives in Psychiatric Care*.

[7] Pashaeypoor S., Baumann S. L., Sadat Hoseini A., Cheraghi M. A., Chenari H. A. (2019). Identifying and overcoming barriers for implementing Watson's human caring science. *Nursing Science Quarterly*.

[8] Shin D. H., Ryu W. Y., Jung J. H. (2020). The effect of absorbable and non-absorbable scleral suture on strabismus surgery in the rabbits. *Current Eye Research*.

[9] Peng L., Liu Y. H., He S. X., Di X. P., Shen H., Luo D. Y. (2020). Is absorbable suture superior to permanent suture for uterosacral ligament suspension. *Neurourology and Urodynamics*.

[10] Yao L., Dolo P. R., Shao Y. (2020). Absorbable suture can be effectively and safely used to close the mesenteric defect in a gastric bypass Sprague-Dawley rat model. *BMC Surgery*.

[11] Liu S., Wang Y., Kotian R. N. (2018). Comparison of nonabsorbable and absorbable suture in total knee arthroplasty. *Medical Science Monitor*.

[12] Matthews C. A., Geller E. J., Henley B. R. (2020). Permanent compared with absorbable suture for vaginal mesh fixation during total hysterectomy and sacrocolpopexy: a randomized controlled trial. *Obstetrics and Gynecology*.

[13] Wallace D. K., Christiansen S. P., Sprunger D. T. (2018). American academy of ophthalmology preferred practice pattern. *Ophthalmology*.

[14] Zeuchner J., Graf J., Elander L., Frisk J., Fredrikson M., Chew M. S. (2021). Introduction of a rapid sequence induction checklist and its effect on compliance to guidelines and complications. *Acta Anaesthesiologica Scandinavica*.

[15] Topalel S., Orekici Temel G., Azizoğlu M. (2020). Evaluation of preoperative anxiety in Turkish paediatric patients and validity and reliability of the Turkish modified Yale preoperative anxiety scale. *Turkish Journal of Anaesthesiology and Reanimation*.

[16] Fadayevatan R., Alizadeh-Khoei M., Hessami-Azar S. T., Sharifi F., Haghi M., Kaboudi B. (2019). Validity and reliability of 11-face faces pain scale in the Iranian elderly community with chronic pain. *Indian Journal of Palliative Care*.

[17] Zhang W., Qi S., Zhuo J., Wen S., Fang C. (2020). Concordance study in hepatectomy recommendations between Watson for oncology and clinical practice for patients with hepatocellular carcinoma in China. *World Journal of Surgery*.

[18] Fox B. I. (2019). Cognitive computing and Watson: implications for hospital pharmacy. *Hospital Pharmacy*.

[19] Paduca A., Arnaut O., Beschieru E., Lundmark P. O., Bruenech J. R. (2021). Shared decision making and patients satisfaction with strabismus care-a pilot study. *Bmc Medical Informatics and Decision Making*.

[20] Dembinski R. L., Collins M. E., Kraus C. L. (2019). Outcomes following surgery for horizontal strabismus in children of lower socioeconomic backgrounds. *Strabismus*.

[21] Wang Y. H., Lee M. C. (2019). Nursing experience using Watson's caring theory to mitigate suicidal behaviors in a homosexual male. *Hu li za zhi The Journal of Nursing*.

[22] Gürcan M., Atay Turan S. (2021). Examining the expectations of healing care environment of hospitalized children with cancer based on Watson's theory of human caring. *Journal of Advanced Nursing*.

[23] Estes K. J., Parrish R. K., Sinacore J., Mumby P. B., McDonnell J. F. (2020). Effects of corrective strabismus surgery on social anxiety and self-consciousness in adults. *Journal of American Association for Pediatric Ophthalmology and Strabismus*.

[24] Karstädt N., Crozier T. A., Horn M., Naxer S., Schittkowski M. P. (2020). Postoperative behaviour after primary strabismus surgery in children: is there an influence of intraoperative topical anaesthesia. *Klinische Monatsblätter für Augenheilkunde*.

[25] Cho J., Kim H. J., Lee J. S. (2020). Comparing absorbable and nonabsorbable suture materials for repair of Achilles tendon rupture: a magnetic resonance imaging-based study. *Diagnostics*.

[26] Kowalski J. T., Genadry R., Ten Eyck P., Bradley C. S. (2021). A randomized controlled trial of permanent vs absorbable suture for uterosacral ligament suspension. *International Urogynecology Journal*.

[27] Promelle V., Aroichane M. (2020). Large muscle cyst following use of non-absorbable suture for strabismus surgery. *Journal of Pediatric Ophthalmology and Strabismus*.

